This article has been retracted.

# First report of the Phe1534Cys *kdr* mutation in natural populations of *Aedes albopictus* from Brazil

**DOI:** 10.1186/s13071-017-2089-5

**Published:** 2017-03-27

**Authors:** Oscar Alexander Aguirre-Obando, Ademir Jesus Martins, Mário Antônio Navarro-Silva

**Affiliations:** 1 Laboratório de Entomologia Médica e Veterinária, Setor de Ciências Biológicas, Departamento de Zoologia, Universidade Federal do Paraná, PO Box 19020, Curitiba, 81531-980 Paraná Brazil; 2 Laboratório de Fisiologia e Controle de Artrópodes Vetores, Instituto Oswaldo Cruz-FIOCRUZ, Av. Brasil 4365, Rio de Janeiro-RJ, PO Box 2104-900, Brazil; 3 Instituto Nacional de Ciência e Tecnologia em Entomologia Molecular, Rio de Janeiro, RJ Brazil

**Keywords:** Allele-specific PCR, Chikungunya, Dengue, Pyrethroid resistance, Vector control, Voltage-gated sodium channel, Zika

## Abstract

**Background:**

Knockdown resistance (kdr), caused by alterations in the voltage-gated sodium channel (Na_V_), is one of the mechanisms responsible for pyrethroid (PY) resistance. In the Asian tiger mosquito, *Aedes albopictus*, at least four different mutations were described in the IIIS6 Na_V_ segment in populations from Asia, North America and Europe. In contrast, in *Aedes aegypti* at least 12 non-synonymous mutations have been reported at nine different codons, mostly in the IIS6 and IIIS6 Na_V_ segments. The Phe1534Cys *kdr* mutation in the IIIS6 Na_V_ segment is the most prevalent in populations of *Ae. aegypti* worldwide, also found in *Ae. albopictus* from Singapore. Herein, we investigated the DNA diversity corresponding to the IIS6 and IIIS6 Na_V_ segments in natural populations of *Ae. albopictus* from Brazil.

**Methods:**

DNA from eight Brazilian *Ae. albopictus* natural populations were individually extracted and pooled by states of origin, amplified, cloned and sequenced for the corresponding IIS6 and IIIS6 Na_V_ segments. Additionally, samples from each location were individually genotyped by an allelic specific PCR (AS-PCR) approach to obtain the genotypic and allelic frequencies for the 1534 Na_V_ site.

**Results:**

No non-synonymous substitutions were observed in the IIS6 sequences. However, the Phe1534Cys *kdr* mutation was evidenced in the *Ae. albopictus* Na_V_ IIIS6 segment sequences from Paraná (PR) and Rondônia (RO) states, but not from Mato Grosso (MT) state. The 1534Cys^*kdr*^ allele varied from 3% (Marilena/PR and Porto Velho/RO) to 10% (Foz do Iguaçu/PR). To our knowledge, this paper reports the first occurrence and provides distribution data of a possible *kdr* mutation in *Ae. albopictus* in South America.

**Conclusion:**

The emergence of a likely *kdr* mutation in *Ae. albopitus* natural populations is a signal of alert for vector control measures since PY are the most popular insecticides adopted by residents. Additionally, once the *kdr* allele is present, its frequency tends to increase faster under exposition to those compounds. Although the Asian tiger mosquito is not incriminated as an important vector of dengue, chikungunya and Zika viruses in South America, its importance in this regard has been extensively discussed since *Ae. albopictus* is rapidly spreading and can also migrate between sylvatic and urban environments. Therefore, insecticide resistance monitoring initiatives should also be extended to *Ae. albopictus* in Brazil in order to maintain chemical compounds as an efficient vector control tool when needed.

**Electronic supplementary material:**

The online version of this article (doi:10.1186/s13071-017-2089-5) contains supplementary material, which is available to authorized users.

## Background

The Asian tiger mosquito, *Aedes albopictus* (Skuse, 1894), presents vector competence for 26 arboviruses, playing an important role in the transmission of dengue, chikungunya and Zika viruses as well as filarial nematodes in Asia and Africa [1–7]. So far, *Ae. aegypti*, a species that shares ecological niches with *Ae. albopictus* [8], is the primary vector for these arboviruses in the Americas [9–11]. However, the vectorial capacity/competence of the Asian tiger mosquito in the two continents has been intensively discussed [4, 5, 12–14]. In South America, *Ae. albopictus* was detected for the first time in Brazil (São Paulo state) in 1986 [15] and is currently present in 24 of the 27 Brazilian federal units, around 59% of all municipalities [16].

Several studies are ongoing in order to develop a vaccine against these arboviruses [17, 18], but the current means of control still relies upon vector control population densities: ideally first targeting the elimination of larval breeding site sources and, secondly insecticide application, which has been many times employed as the principal component of vector control strategies [19]. As a consequence, the intense use of these compounds by both the governmental campaigns and citizens (i.e. constant and uncontrolled household self-application) has been selecting resistant populations to practically all classes of insecticides available in public health [20]. Four classes of neurotoxic insecticides, organochlorines (OC), carbamates (CA), organophosphates (OP) and pyrethroids (PY), have been successively enlisted since the 1950s to control mosquito populations [21].

In contrast to *Ae. aegypti*, few reports of insecticide resistance in *Ae. albopictus* are known. Globally, this lack of information about the insecticide resistance status of *Ae. albopictus* is obviously related to its less significant role in arbovirus disease transmition in most of the world, compared to *Ae. aegypti* [22]. However, attention to the control of the Asian tiger mosquito should not be neglected even when both species are present since *Ae. albopictus* is a main connection between sylvatic/rural and suburban landscapes [23]. So far, some PY and one OP are recommended by WHO Pesticide Evaluate Scheme (WHOPES) for adult population vector control programmes [24]. Worldwide, PY are the most common class of insecticides to control adult vector-borne diseases due to their rapid effect (knockdown, similar to DDT) and safety [25]. As a consequence, there are plenty of resistance registers against PY in *Aedes* and *Anopheles* mosquitoes [26, 27], including some *Ae. albopictus* populations [20, 22, 28, 29].

Metabolic alterations and target site insensitivity represent the two major forms of PY resistance [30]. Pyrethroids and OC (DDT) target the voltage-gated sodium channel (Na_V_) in insects, producing an effect similar to a knockdown [31]. This channel is a transmembrane protein present in the neuronal axons, composed of four homologous domains (I-IV), each with six hydrophobic segments (S1-S6) [32]. Several point mutations were reported in Na_V_ insects, most of which in the IIS6 and IIIS6 Na_V_ segments very well related to PY resistance, known as *kdr* mutations [33, 34]. In *Ae. aegypti*, several *kdr* mutations were identified, especially at the Na_V_ positions 989, 1011 and 1016 (IIS6 segment) as well as 1534 (IIIS6 segment) [35–38]. In *Ae. albopictus*, however, only four alterations were found, at the 1532 and 1534 positions, both in the IIIS6 segment. The Phe1534Cys *kdr* mutation, similar to the most frequent *kdr* mutation in *Ae. aegypti*, was reported in Singapore [39], China [40] and Greece [41]; 1534Leu in the USA [42] and China [40, 41]; and 1534Ser also in the USA and China [41]. The substitution at the 1532 position (Ile1532Thr) appeared only in the *Ae. albopictus* population from Italy [41].

Given the increasing dispersion of *Ae. albopictus* and the possible role of this insect in the maintenance or even transmission of dengue, chikungunya and Zika viruses, this study was undertaken to investigate the occurrence, frequency and distribution of possible *kdr* mutations eventually, discovered in the IIS6 and IIIS6 Na_V_ segments in Brazilian *Ae. albopictus* natural populations. Herein, we identify the existence of the Phe1534Cys *kdr* mutation in natural *Ae. albopictus* populations from Brazil.

## Methods

### Sampling

The collection of *Aedes* spp. from the municipalities of Cianorte, Foz do Iguaçu, Maringá, Marilena, Nova Londrina, Alvorada do Sul (Paraná state), Rondonópolis (Mato Grosso state) and Porto Velho (Rondônia state) followed the instructions of the Brazilian *Ae. aegypti* Insecticide Resistance Monitoring Network (MoReNAa) [43]. Geopolitically, Paraná, Mato Grosso and Rondônia states are part of the South, Central-West and North regions, respectively. Geographical locations as well as years of sampling are represented in Fig. 1. All samples were collected by the dengue vector control programme staff members from each municipality. In all cases ovitraps were installed at least 100 m apart in the peridomestic area [44]. The samples collected were sent to the Medical Entomology and Veterinary Laboratory of Parana Federal University. The gathered *Aedes* spp. eggs were induced to hatch in the laboratory and reared until adult emergence under controlled conditions (25 ± 1 °C, humidity 80 ± 10% and photoperiod 12:12 h). These adult mosquitoes from each population were species identified following the identification keys of Consoli et al. [45] and Forattini [46]. Recently-emerged *Ae. albopictus* adults from each population were collected for molecular analysis. The mosquitoes were individually placed in absolute ethanol (99.5%) and stored at -20 °C.

**Fig. 1:** Allelic frequencies for the 1534 Na_V_ *kdr* site of *Aedes albopictus* from Brazil. Cities/States of collection and the year of sampling (in parentheses) are placed in the map. Paraná state is detached, showing its multiple cities of collection

### Amplification, cloning and sequencing of the IIS6 and IIIS6 Na_V_ segments of *Ae. albopictus*

DNA extraction followed Aguirre-Obando et al. [47] guidelines. All the samples from each locality were individually extracted. The amount of 1 μl [20 ng/μl] of each extraction was added to form a DNA pool for each of the three states: Paraná (*n* = 118), Mato Grosso (*n* = 11) and Rondônia (*n* = 37). These DNA pools were used to amplify the genomic region correspondent to the IIS6 and IIIS6 Na_V_ segments, as proposed elsewhere [36, 48]. The employed primers had been previously designed for *Ae. aegypti*: 5para3 (5′-ACA ATG TGG ATC GCT TCC C-3′) and 3para3 (5′-TGG ACA AAA GCA AGG CTA AG-3′) [48], and AaEx31P (5′-TCG CGG GAG GTA AGT TAT TG-3′) and AaEx31Q (5′-GTT GAT GTG CGA TGG AAA TG-3′) [36], respectively, for the IIS6 and IIIS6 Na_V_ segments. Notably, the Na_V_ sequences present high similarity between *Ae. aegypti* and *Ae. albopictus*, and the region of primers annealing were identical.

Polymerase chain reactions (PCR) amplifications were carried out with the USB® FideliTaq™ DNA Polymerase kit (Affymetrix; 0.03 U Taq DNA polymerase and 1× buffer) containing 20 ng/μl of the genomic DNA pool, 1 μM of each primer and 0.25 μM of dNTP in 40 μl of reaction. PCR conditions for both IIS6 and IIIS6 Na_V_ segments were: 95 °C for 5 min, followed by 35 cycles of 95 °C for 30 s, 60 °C for 40 s and 72 °C for 1 min with a final extension step at 72 °C for 5 min. The PCR products were purified using the magnetic beads approach (Agencourt® AMPure® XP, Beckman Coulter, Inc.) from which 2 μl were applied to carry out the ligation reaction with the CloneJet PCR Cloning Kit (Thermo Scientific, Pittsburgh, USA), both in accordance with the manufacturer’s instructions. The volume of 3 μl from the ligation reaction was used to transform *Escherichia coli* DH5α competent cells. Around 200 randomly chosen colonies were inoculated in 1 ml of Circlegrow medium (MP Biomedicals, Santa Ana, USA) with 1 mg/l ampicillin in deep well plates and then incubated for 22 h at 37 °C and 220 rpm. The DNA minipreps followed the alkaline lysis procedure [49]. The sequencing reactions were performed with the Big Dye 3.1 Kit (LifeTechnologies/Applied Biosystems, California, USA), in compliance with the manufacture’s instructions, and sequenced on an ABI377 automated sequencer (LifeTechnologies/Applied Biosystems, California, USA) in the DNA sequencing facility of FIOCRUZ (Plataforma de Sequenciamento/PDTIS/Fiocruz).

Sequence analyses were performed with the software Geneious® (R7.1.3. Biomatters, Auckland, New Zealand) and the Blast platform of NCBI. Only changes in sequences of at least two independent clones were considered, as some of the singletons might represent PCR-induced mutations [48]. The haplotypes in this study were deposited in the GenBank database (accession numbers KX281169–KX281170 and KX371864–KX371865). Mega 6.1 [50] software was used to translate the IIS6 and IIIS6 segments into amino acid sequences to check for the existence of non-synonymous mutations. The codon numeration was determined in accordance with *Musca domestica* Na_V_ numbering.

### Genotyping of the 1534 Na_V_ site of *Ae. albopictus*

Given the high conservation at the genomic Na_V_ sequence coding for the IIIS6 segment between *Ae. aegypti* and *Ae. albopictus*, we employed the same allele-specific PCR assay (AS-PCR) previously designed for the Phe1534Cys variation in *Ae. aegypti* [36]. In this reaction three primers were engaged, one reverse common for both alleles: 5′-TCT GCT CGT TGA AGT TGT CGA T-3′, and two forward allele specific primers: 1534Phe^+^: 5′-GCG GGC TCT ACT TTG TGT TCT TCA TCA TAT T-3′ and 1534Cys^*kdr*^ allele: 5′-GCG GGC AGG GCG GCG GGG GCG GGG CCT CTA CTT TGT GTT CTT CAT CAT GTG-3′. Briefly, the discrimination of the PCR products was possible due to a GC tail attached to the 5′-end of the primers, differing in 20 nucleotides between them. Additionally, an increase in the specificity of the reaction was obtained by a transversion in the antepenultimate nucleotide at 3′-end of each allelic specific primer [38, 51, 52]. Around 15 samples from each population were individually genotyped following the protocol described by Linss et al. [37]. All batches of reactions included positive controls for the genotypes 1534 Phe/Phe, Cys/Cys and Phe/Cys, taken from DNA of the *Ae. aegypti* lineages, respectively Rockeffeller (Rock), Rock-*kdr* and a mix of them in equimolar concentrations. The *Ae. aegypti* Rockefeller lineage is a standard for vigor and insecticide susceptibility [53], whilst the Rock-*kdr* is a PY resistant lineage, previously selected in our laboratory for both 1016Ile^*kdr*^ and 1534Cys^*kdr*^ mutations in the Na_V_ (for more details see: Brito et al. [54]). The AS-PCR amplicons were evaluated in 10% polyacrylamide electrophoresis gel stained in a Safer dye solution bath (Kasvi: 6×). By analyzing the amplicons, the genotype and allelic frequencies were calculated and the Hardy-Weinberg equilibrium (HW) hypothesis test was carried out [55]. These analyses were conducted in two different ways: first, each municipality was considered and analyzed individually and second, the municipalities from Paraná state were pooled and analyzed together.

## Results

In the total sampling, *Ae. albopictus* represented an average of 6.4% of the eggs collected, the remaining being *Ae. aegypti*. Table 1 shows some demographic information and the total number of adult mosquitoes obtained from each locality. The yearly number of dengue cases for these municipalities is presented in Additional file 1: Table S1. The locality with the lowest prevalence of *Ae. albopictus* (1.3%) was Foz do Iguaçu which is also the city with the fewest inhabitants living in a rural area (0.8%). Accordingly, higher prevalence of *Ae. albopictus* was, in general, observed in the cities with higher human densities in the rural area.

**Table 1:** Demographic data and numbers of *Aedes aegypti* and *Aedes albopictus* in the localities studied

Municipality	Demographic information^a^				Sampling^b^		
	Inhabitants	Residents in rural area (%)	Area (km^2^)	Inhabitants/km^2^	Year of sampling	*Ae. aegypti*	*Ae. albopictus*
Porto Velho (RO)	428,527	8.8	34,090.9	12.6	2010	9,203	162 (1.7%)^c^
Rondonópolis (MT)	195,476	3.8	4,159.1	47.0	2012	1,383	23 (1.6%)
Nova Londrina (PR)	13,067	8.1	269.4	48.5	2014	236	21 (8.2%)
Alvorada do Sul (PR)	10,283	28.6	424.3	24.2	2014	219	17 (7.2%)
Cianorte (PR)	69,958	11.0	811.7	86.2	2009	1,181	262 (18.2%)
Marilena (PR)	6,858	27.3	232.4	29.5	2014	143	16 (10.1%)
Foz do Iguaçú (PR)	256,088	0.8	618.4	414.1	2009	5,544	73 (1.3%)
Maringá (PR)	357,077	1.8	487.1	733.1	2012	13,436	393 (2.8%)

*Abbreviations: MT* Mato Grosso State, *RO* Rondonia State, *PR* Paraná State

^a^Source: IBGE Cidades, 2010 sense (http://www.cidades.ibge.gov.br/)

^b^Adult mosquitoes reared in laboratory conditions resulting from the eggs collected in the field

^c^ % of *Ae. albopictus* among total *Aedes* mosquitoes

The genomic region corresponding to the IIS6 (294 bp) and IIIS6 (350 bp) Na_V_ segments of *Ae. albopictus* from three Brazilian states, Rondônia (North region), Mato Grosso (Central-West region) and Paraná (South region), were obtained, amplified and sequenced from a total of 166 mosquitoes. A total of 96 sequences of the IIS6 Na_V_ segment displayed two distinct haplotypes, differing in only one nucleotide insertion in the intronic region (GenBank: KX281169 and KX281170). Both haplotypes, IIS6_H1 (52.6%) and IIS6_H2 (47.4%), were detected in clones representative of all states (Table 2). Figure 2 shows an alignment of the IIS6 haplotypes reported herein, three genomic sequences of *Ae. albopictus* available in the GenBank database, from Brazil (FJ479615), Malaysia (KC152045) and Japan (AB827810) as well as one *Ae. aegypti* haplotype from Brazil (FJ479611), evidencing a high similarity. None of the haplotypes presented non-synonymous substitutions (Fig. 2).

**Table 2:** Distribution and frequency of the IIS6 and IIIS6 Na_V_ haplotypes of *Aedes albopictus* from Brazil. The frequencies considered the total amount of clones from the respective IIS6 or IIIS6 segments

Haplotype	Haplotype frequency (%)			Total
	Paraná	Mato Grosso	Rôndonia	
IIS6 H1	36.7	5.3	10.6	52.6
IIS6 H2	34.2	4.0	9.2	47.4
IIIS6 1534Phe	41.7	12.5	21.9	76.1
IIIS6 1534Cys	20.8	0.0	3.1	23.9

**Fig. 2:** Nucleotide diversity in the IIS6 Na_V_ segment of *Aedes albopictus*. ClustalW alignment for comparing the haplotypes found in this study, IIS6_Hap1 (KX281169) and IIS6_Hap2 (KX281170), with other sequences of *Ae. albopictus* available in GenBank from Brazil (FJ479615), Malaysia (KC152045) and Japan (AB827810). One haplotype of *Ae. aegypti* (FJ479611) was included for comparison, but the intron was neglected in order not to disturb the alignment. The sequence AB827810 does not cover the whole extension of this alignment. The translated amino acid sequence is represented by the letters in *blue*, over the first nucleotide of their corresponding codon. Nucleotides in uppercase letters correspond to the coding region (exons 20 and 21), and those in lower case refer to the intron with the numbering in the alignment inside brackets at the top of each block and underlined sequences referring to the primers positions. Invariable sites are indicated with dots, otherwise with the alternative nucleotide and gaps with (-). Squares indicate the codons where the 989, 1011 and 1016 *kdr* mutation sites are present in *Ae. aegypti*

Regarding the IIIS6 Na_V_ segment, from 96 clone sequences, two haplotypes were also detected in which the only polymorphism was the single nucleotide polymorphism (SNP) TTC/TGC, corresponding to the known Phe1534Cys *kdr* mutation. The 1534Cys^*kdr*^ haplotype was present in the IIIS6 clones of *Ae. albopictus* from Paraná (20.8%) and Rondônia (3.1%) states but not from Mato Grosso state (Table 2). These sequences were also submitted to the GenBank (KX371864 and KX371865). Figure 3 shows an alignment of the IIIS6 haplotypes and some of the few homologous regions available in the GenBank for *Ae. albopictus*, one DNA (AB827824) and two mRNA sequences (KC152046 and AY663382), none of them covering the whole extension of our sequences. A homologous *Ae. aegypti* sequence (KF527415) was also added to the alignment, demonstrating that the AS-PCR primers developed for the 1534 Na_V_ site of this species is also suitable for these Brazilian *Ae. albopictus* populations.

**Fig. 3:** Nucleotide diversity in the IIIS6 Na_V_ segment of *Aedes albopictus*. ClustalW alignment for comparing the haplotypes found in this study, 1534Phe (KX371864) and 1534Cys (KX371865), with other *Ae. albopictus* sequences available in GenBank: genomic DNA (AB827824), mRNA (KC152046 and AY663382) and one haplotype of *Ae. aegypti* (KF527415). The three sequences downloaded from GenBank do not cover the whole extension of this alignment. The translated amino acid sequence is represented by the letters in blue, over the first nucleotide of their corresponding codon. Nucleotides in uppercase letters correspond to the coding region (exons 30 and 31) and those in lower case refer to the intron, with the numbering in the alignment inside brackets at the top of each block and single underlined sequences referring to the primers positions. Double underlines indicate the annealing region for the AS-PCR primers. Invariable sites are indicated with dots, otherwise with the alternative nucleotide and gaps with (-). The 1534 *kdr* site is indicated with a square

Once the Phe1534Cys *kdr* mutation was evidenced in our samples, we evaluated the allelic and genotype frequencies from each municipality for the 1534 *kdr* site. The 1534Cys^*kdr*^ allele ranged from 0 to 10% amongst the six municipalities of Paraná state, 3% in Porto Velho (Rondônia state) and was not present in Rondonópolis (Matto Grosso state) (Fig. 1). In all cases, when the *kdr* allele was found, it appeared in heterozygosis with no rejection of the HW Equilibrium hypothesis in any case (*P* > 0.05) (Table 3).

**Table 3:** Genotype frequency of the 1534 Na_V_ site of eight *Aedes albopictus* population from Brazil

Location	Year	*N*	Genotype frequency			HWE^a^	
			Phe/Phe	Phe/Cys	Cys/Cys	*χ* ^2^	*P*
Porto Velho (RO)	2010	37	0.95	0.05	0	0.002	0.821
Rondonópolis (MT)	2012	11	1	0	0	–	–
Cianorte (PR)	2009	16	1	0	0	–	–
Foz do Iguaçu (PR)	2009	24	0.79	0.21	0	0.324	0.875
Maringá (PR)	2012	24	0.87	0.13	0	0.107	0.753
Marilena (PR)	2014	16	0.94	0.06	0	0.017	0.874
Nova Londrina (PR)	2014	21	1	0	0	–	–
Alvorada do Sul (PR)	2014	17	1	0	0	–	–
PR	2009–2014	118	0.92	0.08	0	0.185	0.768

*Abbreviations: MT* Mato Grosso State, *PR* Paraná State, *RO* Rondonia State

^a^Hardy-Weinberg Equilibrium: Chi-square test with 1 degree of freedom

## Discussion

A very informative compilation of worldwide insecticide resistance data for vector mosquitoes had been published in 1986 [56]. In this review, native *Ae. albopictus* populations from Asia already presented resistance to the OC adulticides, DDT and dieldrin (not currently used in vector control programmes), the OP malathion adulticide and the fenthion larvicide. From 2010 on, new reviews have been focusing on insecticide resistance data on the “dengue vectors” *Ae. aegypti* and *Ae. albopictus* [20, 22, 57]. Among these reviews, out of more than 100 evaluated papers only 35 considered *Ae. albopictus*, in which resistance to OC, OP (larvicide temephos) and PY was registered in some countries from Asia, Africa, Caribbean and Europe. In South America, especially in Brazil, to our knowledge, only one study has evidenced loss of susceptibility to an insecticide, in this case the larvicide OP temephos in *Ae. albopictus* [58].

The *kdr* mutations are highly related to PY resistance in several insect species, including vector mosquitoes, and have been therefore adopted as molecular markers for rapid screening of field populations [33, 59]. To our knowledge, we report here for the first time the Phe1534Cys substitution in the Na_V_ of *Ae. albopictus* in Brazil. Among the four municipalities where the Phe1534Cys *kdr* mutations were found, Porto Velho, Maringá and Foz do Iguaçu are large urban centers with high incidence of dengue outbreaks [60–62]. Foz do Iguaçu deserves special attention since it borders Puerto Iguazú (Argentina) and Ciudad del Este (Paraguay). Although we only have data evidencing loss of susceptibility to the OP Temephos larvicide in Brazilian *Ae. albopictus* populations [58], resistance to both OP and PY was detected in *Ae. aegypti* from Foz do Iguaçu [58, 62]. This indicates strong selection pressure due to the OP and PY insecticides in that locality which is also likely affecting *Ae. albopictus*. A similar mutation was previously described in populations from Singapore [39], China [40] and Greece [41]. In this same 1534 position other alterations were described, 1534Leu and 1534Ser in the USA [41, 42] and China [40, 41]. In a study on *Ae. albopictus* populations from the USA, the status of resistance was confirmed for both OC DDT and OP malathion, but not for the PYs (deltamethrin, phenothrin and prallethrin) although the Phe1534Leu mutation was present [42]. This same mutation could not be correlated to PY resistance in Chinese *Ae. albopictus* populations resistant to the PY deltamethrin. On the other hand, the frequency of Phe1534Ser was significantly higher in the resistant populations than in those found susceptible [41].

Phe1534Cys is the most frequent *kdr* mutation in *Ae. aegypti* populations worldwide and its role to PY resistance is very well defined alone or in conjunction with other Na_V_ mutations [63]. Although we do not have reports of insecticide resistance in *Ae. albopictus* in Brazil, we are aware of the intense selection pressure with these chemical compounds in the country. This is well indicated by the increase in the frequency and spread of *kdr* mutations in *Ae. aegypti*, well related with the intense use of PY in the last decade [37, 64]. The frequency of the 1534Cys^*kdr*^ allele in Brazilian *Ae. albopictus* populations (ranging from 3 to 10%, when found) was low when compared to the findings in Singapore (73%), for instance [39]. Additionally, in our study all insects bearing this mutation were heterozygotes. Anyway, as there was no support for rejecting the HW equilibrium hypothesis, we have no evidence to suggest a possible positive selection for the 1534Cys^*kdr*^. In contrast, some *Ae. albopictus* populations from China and Greece were not under HW equilibrium regarding the 1534 Na_V_ position, probably due to a heterozygote deficit [41]. As low frequencies of the 1534Cys^*kdr*^ were found in our study, and considering that there is a selection pressure with PY favoring the homozygous *kdr* [54] in the studied localities, we suggest that this mutation has just emerged or was introduced very recently in Brazil.

Further phylogenetic analyses incorporating the IIIS6 segment sequences and neutral markers for *Ae. albopictus* from different parts of the world may help explain whether the Phe1534Cys *kdr* mutation arose independently in Brazil or migrated from elsewhere. So far, there are few Na_V_ sequences of *Ae. albopictus* available. Unfortunately, the publications that described *kdr* mutations in the Asian tiger mosquito had not deposited their sequences in GenBank [39–42] up to the date when our study was submitted. Actually, there are 14 sequences with part of the IIIS6 Na_V_ segment of Japanese populations (AB827815–AB827828) (Kawada & Pujiyati, published on GenBank only) but without the intron region, which would be valuable for phylogenetic analysis. More data are needed in order to process such analyses with worldwide samples to infer the origin and dispersion of the *kdr* mutations.

The AS-PCR approach for detecting the presence and frequency of *kdr* mutations is suitable as one of the tools for PY resistance surveillance in natural *Ae. albopictus*. However, prior to carry on this strategy, it is necessary to be aware of the nucleotide diversity in the sequence of the *Na*_*V*_ gene of local populations. A recent survey of *Ae. albopictus* from several countries, in North America, Europe and Asia, reported that the 1534 Na_V_ position is highly variable due to the presence of different mutations such as: TTC and TTT (Phe) as well as the TGC (Cys), TCC (Ser) and TTG (Leu) [40]. This means that one has to know exactly which alleles in the target population exist before applying an AS-PCR approach, like the one herein. We employed specific primers previously designed for the 1534Phe^+^ (TTC) and 1534Cys^*kdr*^ (TGC) alleles [36], after having evidenced sequenced clones of the IIIS6 segments from Brazilian populations of several localities. Another mutation, two positions upstream from the 1534 site (Ile1532Thr), was found in an *Ae. albopictus* population from Rome, Italy [41].

It is important to mention that the amount of *Ae. albopictus* collected in our study might be underestimating the real proportion of this species since the methodologies of vector surveillance by ovitraps are based on *Ae. aegypti* eg-laying preferences. As *Ae. albopictus* prefers conditions with more vegetation and is generally more exophilic than *Ae. aegypti* [65], our samplings may not cover some environments where *Ae. albopictus* is more common. In Brazil, the most recent national survey on *Ae. albopictus* distribution considering the annual larval surveys from 2007 to 2014, displayed that the house infestation index (HI) for *Ae. aegypti* is traditionally higher than that for *Ae. albopictus*. Nevertheless, from 2007 to 2011 in at least 34 municipalities, the HI ratio values for *Ae. albopictus* (median: 1.4) were higher than those for *Ae. aegypti* [16].

Although *Ae. albopictus* is not incriminated as a dengue, chikungunya or Zika virus vector in South America, it shares ecological niches with *Ae. aegypti* in urban areas, therefore suffering the same chemical selection pressure [16]. Thus, the 1534Cys^*kdr*^ allele in this study might have been favorably selected by the constant PY applications in ultralow volume oriented by the Brazilian Dengue Control Programme from 2001 to 2009 [43]. Similar consequences to the PY resistance together with an increase and spread of *kdr* alleles throughout North and South American *Ae. aegypti* populations [37, 47, 66, 67], may take place with *Ae. albopictus* as well. Bioassays with field populations, considering distinct genotypes in the *Na*_*V*_ gene, must be performed in order to confirm the susceptibility status and the role of these variants in PY resistance.

## Conclusions

The presence of a *kdr* mutation in natural *Ae. albopictus* populations from distinct regions of Brazil points to the need of special attention also to this species in relation to insecticide resistance monitoring purposes. New alternative tools are now under implementation for *Ae. aegypti* control in Brazil, such as strains infected with *Wolbachia* and transgenic sterile lines, aiming respectively, to suppress local mosquito populations [68] or replacement by a lineage refractory to arbovirus infection and transmission [69]. If *Ae. albopictus* develops the arbovirus transmission role now assumed for *Ae. aegypti*, it could take its epidemiological place since the Asian tiger mosquito is largely disseminated throughout the country. Therefore, integrated vector control approaches and consistent insecticide resistance monitoring programmes are of prime concern in order to control diseases caused by arboviruses.

## Additional file

Additional file 1: Table S1. Number of dengue cases registered in the localities studied. (DOCX 18 kb)

## Abbreviations

AS-PCR: Allelic specific PCR
HI: Infestation index
HW: Hardy-Weinberg equilibrium
*Kdr*: Knockdown resistance gene
LI: House-to-house larval survey
LIRAa: Rapid assessment of infestation by *Aedes aegypti*
MoReNAa: Brazilian *Aedes aegypti* Insecticide Resistance Monitoring Network
Na_V_: Voltage-gated sodium channel
PY: Pyrethroids
SNP: Single nucleotide polymorphism
